The article "Review on Characterization, Properties, and Analytical Methods of Cefepime" was published in 2022. Journal: Int J Anal Chem.

# Review on Characterization, Properties, and Analytical Methods of Cefepime

**DOI:** 10.1155/2022/6909528

**Published:** 2022-06-29

**Authors:** Omkulthom Al kamaly

**Affiliations:** Department of Pharmaceutical Sciences, College of Pharmacy, Princess Nourah Bint Abdulrahman University, P.O. Box 84428, Riyadh 11671, Saudi Arabia

## Abstract

Infection is one of the most important reasons for the increase in the number of deaths worldwide; it can be a bacterial or viral infection. As a result, there are many effective drugs against this infection, especially bacterial ones. Cefepime (CP) is one of the fourth generations of cephalosporins and is distinguished from others in that it can kill both positive and negative bacteria. Therefore, this study focused on the chemical properties of the drug, its uses, and its stability against bacteria. All analysis methods for this drug in pharmaceutical preparations, blood, or plasma were also presented. One of the important problems in these methods is using toxic solvents, which poses a danger to society and the environment. The presentation of these solvents will allow companies to manufacture and use more effective and less toxic solvents.

## 1. Introduction

Cefepime (CP) is one of the commonly used fourth-generation cephalosporins. Cefpirome and cefaclidine are other fourth-generation antibiotics. CP has adequate *β*-lactamase stability but with a low affinity for extended spectrum. The broad spectrum of CP is imposed to cover a wide range of positively and negatively pathogens [1–4]. Compared with ceftazidime from the fourth generation in vitro, CP has intensified activity against Gram (+) bacteria, excluding the species sensitive to methicillin, such as *Streptococcus pneumoniae* and *Staphylococcus aureus* [5, 6]. CP is more effective against extended-spectrum *β*-lactamase Gram (−) bacteria than other oxyimino-cephalosporins commercially available. [7–9].

The cefepime's chemical structure is displayed in Figure 1. The basic cephem ring at position 7 is modified chemically to increase the cephalosporins' stability against *β*-lactamase enzymes. Similarly, other antibiotics CP such as ceftazidime, cefoperazone, ceftizoxime, and ceftriaxone from the third-generation contain a 2-amino thiazolyl acetamido group substituted with an oxyimino in the same position. However, unlike other third-generation cephalosporins, CP possesses a cephem nucleus substituted with a positively charged NMR, making it a zwitterion [2]. This zwitterionic property permits penetration of CP to Gram (+) bacteria's porin channels rapidly [10, 11]. CP is used effectively to treat severe urinary and respiratory tract infections, as well as infections of the skin, soft tissues, and the women's reproductive tract among patients with febrile neutropenia. Treatment of pneumonia in cystic fibrosis patients with this medication is superior to that with ceftazidime.

CP is considered an empirical monotherapy for pneumonia; it is widely used currently in hospitals for this approved indication and given to the patient with abdominal, urinary tract, febrile neutropenia, and skin or soft tissue infections. An earlier systematic published review of empirical monotherapy for the treatment of febrile neutropenia found CP to be associated with a higher mortality rate than other *β*-lactam antibiotics. It was unclear how the higher mortality rate was explained. CP was associated with more superinfections than other *β*-lactams, though the difference was not significant statistically. [12]. The authors in [1] established that the overall death rate was significantly lower in patients suffering from *P. aeruginosa* infections if treated with extended infusion CP.

## 2. Stability

In aqueous solutions, either acidic or basic, CP undergoes rapid degradation, resulting in hydrolysis (opening) of the *β*-lactam ring and simultaneous release of the side chain in the R-2 position from its particle. Because of hydrolysis of the *β*-lactam ring and separation of the NMP particle, two degradation products have been observed, neither of which demonstrate antimicrobial activity.2-[((2-amino-4-triazolyl) (methoxyimino)acetyl) amino] acetaldehyde is one of them [5]. The rate at which CP degrades in aqueous solutions, just like other *β*-lactam antibiotics, is determined by temperature, light, solvent composition, pH, antibiotic concentration, and the type of packaging. [7].

## 3. Chemistry

Cephalosporins, in general, contain a 4-membered *β*-lactam cycle connected to a 6-membered dihydrothiazine cycle [8]. The molecular weight of CP is 571.5 g, and its molecular formula is C_I9_H_25_N_6_O_5_S_2_·Cl·HCl·H_2_O. CP named chemically as (6R,7R)-7-((E)-2-(2-aminothiazol-4-yl)- 2-(methoxyimino) -acetamido)-3-((1-methylpyrrolidin-1-ium-1-yl) methyl)-8-oxo-5-thia-1-azabicyclo [4.2.0] oct-2-ene- 2-carboxylate, its structure is shown in Figure 1, and it is characterized by high solubility in water. Furthermore, it is supplied as intravenous (IV) and intramuscular (IM) administration in doses equivalent to 2 g, 1 g, and 0.5 g of CP. It is formulated as a hydrochloride salt and used with L-arginine, adjusting the reconstituted solution at pH 4–6. [8].

CP is cited as an antibiotic from the fourth generation because its activity is a broad spectrum, and it has a high resistance to hydrolysis by *β*-lactamase [12]. CP possesses a quaternary positively charged nitrogen atom, thus, it is called a zwitterion. This character makes CP neutral enough and increases its ability to penetrate bacterial membranes [13]. CP has a side chain with a 2-amino thiazolyl acetamido group at position 7 and is substituted with the alpha-oxyimino group. The 2-carboxy-2-propoxyimino group in CP is replaced by the alkoxyimino group at position 7, as is the case with cefotaxime, ceftriaxone, and ceftazidime. [14] This is expected to increase its stability against *β*-lactamases by avoiding the entrance of these enzymes into the nucleus. The antistaphylococcal activity is improved by substituting the group (7-[2-carboxy-2-propoxyimino]) in its side chain with an alkoxyimino substituent. Therefore, CP has a similar gram (−) spectrum and better antistaphylococcal activity than ceftazidime [14].

## 4. Mechanism of Action

The *E. coli* porin channel penetration by CP, cefaclidine, and cefpirome is at least 5–10 times faster than ceftazidime and cefotaxime. CP has stability against plasmid-mediated *β*-lactamase SHV-1 and SHV-2, OXA-1 and OXA-3, PSE-1, and PSE-2, and TEM-1 and TEM-2 [2]. The relative hydrolysis rates correspond to that of cefpirome [15,16], cefotaxime, latamoxef, and ceftazidime but are lesser than cefoperazone. Testing CP against 326 members of the Enterobacteriaceae found that it is more active than moxalactam, cefoperazone, cefotaxime, cefpirome, and ceftazidime. Because CP has a low empathy for the major chromosomally mediated 13-lactamase, it is probably less influenced by the nonhydrolytic barrier mechanism of bacterial resistance. CP may demonstrate to be a powerful therapy for microbial infections that are unaffected by other antimicrobials. For instance, in a new study, CP resistance rarely appeared among cefotaxime and ceftazidime-resistant *Pseudomonas aeruginosa* mutants [17].

## 5. Indications and Side Effects

The use of cefepime for treating UTIs in children has been perceived as safe and effective with the least adverse effects. Considering its broad spectrum of antimicrobial activity, it is a convenient candidate for early empiric curing of critically ill children, especially those who suffer from anatomical abnormalities of the urinary tract in which antibiotic-resistant microbes may be present less commonly [18–20] as well as infections of the skin and skin structure can be treated with CP. Besides treating bacterial infections, CP is used to cure gynecologic and intraabdominal infections, febrile neutropenia, bacteremia, meningitis, and long-term bronchopulmonary infections associated with cystic fibrosis in pediatric patients [8]. The effect of the combination of nacubactam as a *β*-lactamase inhibitor and CP against *Escherichia coli* and *Klebsiella pneumonia,* which are carbapenem-resistant, was reported in [21] by the authors in [22]. Cefepime is highly effective in treating COVID-19 patients with moderate and severe symptoms. Cefepime has a highly antiviral effect and is effective against large-scale viruses, including SARS and MERS. When combined with antibiotics or steroids, cefepime is considered more effective than when taken alone.

There should be a consideration for CP neurotoxicity in older patients with myoclonus who are suffering recently from alterations in mental status and renal impairment [23–26]. Seizures are the most common adverse reaction of cefepime on the central nervous system. It can also cause encephalopathy [27, 28]. Several drugs are known to cause nephrotoxicity, notably beta-lactamase inhibitors, and cephalosporins. Despite a few severe side effects, cefepime is a widely prescribed fourth-generation cephalosporin. Numerous reports suggested that cefepime may produce neurotoxicity, but there is no evidence that it causes acute interstitial nephritis. [29].

## 6. Analytical Methods for Determining CP

It is extremely imperative to quantify CP to manage bioequivalence and bioavailability studies besides pharmacokinetic parameters for curing observation. There are about 58 methods proposed for its analysis, either in pharmaceutical dosage forms, serum, or in plasma. These methods were collected from Google Scholar, PubMed, Web of Science, Scopus, and Science Direct. In this work, determination of CP by reverse phase-HPLC and HPLC, as shown in Table 1, was prevalent. With HPLC techniques, quantitative studies are characterized by the efficiency, specificity, speed, and accuracy with tracking capabilities.  Table 2 contains micellar electrokinetic chromatographic methods. Some potentiometric and electrochemical methods are mentioned in Table 3, while the chromatographic technique is combined with other techniques such as LC, and HPLC. UPLC, MS, and MEKC are cited in Table 4. One of the commonly used techniques was UV absorption spectroscopy, which is used alone or with other techniques and based on colorimetry, fluorometry, and other spectrophotometric methods. All these methods are stated in Table 5.  Table 6 includes gas chromatographic methods. Most of the summarized methods utilized different chemically toxic solvents as shown in all tables. Consequently, it is awfully significant for development and verification to select the analytical methods to be applied to reduce the number of toxic products. This is because it may destroy the environment, the instruments used, and the operators. To minimize such issues, it is imperative to pick an apparatus that is more specific and as sensible as other, which has low costs of analysis and therefore reduces power depletion (a factor that directly affects the last price of an outcome). It needs smaller quantities of solvents or that can recognize lower concentrations, it can retrieve dangerous solvents (in order to reduce the risk of pollution in the surroundings), and it can guide pharmaceutical companies and researchers to consume nontoxic solvents and enhance the habitat to decrease the risk of contamination. Hence, the analysis should take the contribution of universities and research centers into consideration to verify the quality of drugs and their safety in application to the public.

## 7. Conclusions

Cefepime is one of the important drugs from the cephalosporin group as it is distinguished from the rest of the group by its resistance to bacteria, which allows it to work on many positive and negative bacterial pathogens. The drug's stability is due to the chemical modification of its structure in the 7-position of the cephem ring, and the cephem nucleus substituted with a positively charged N-methyl-pyrrolidine, making it a zwitterion. This zwitterionic property permits penetration of the drug to Gram (+) bacteria's porin channels rapidly, so it is used effectively to treat severe urinary and respiratory tract infections. Furthermore, many recent studies have proven its worth in treating cases of skin, soft tissues, and the women's reproductive tract among patients with febrile neutropenia either it is found to be superior in the treatment of pneumonia in cystic fibrosis patients, which drew the attention of many researchers to analyse this drug in several methods in its dosage forms or in plasma or serum, and the most common analysis methods for this drug are HPLC.

## Figures and Tables

**Figure 1:** The zwitterion form of cefepime (CP).

**Table 1:** Detection of CP quantitatively by HPLC methods.

Column (C)	Mobile phase	Flow rate (ml/min)	Wavelength (nm)	Matrices	Reference
Supelcosil ABZ + (5 *μ*m;150 × 4.6 mm)	20 mM PDPB pH 2:ACN (94 : 6, *v*/*v*, *v*/*v*).	1	263	Human serum	[30]
Hypersil BDS C18	Acetate buffer pH 4:ACN (97.2 : 2.8 *v*/*v*)	1	254	Human plasma	[31]
Hypersil BDS C18	MeOH:25 mM SDPM pH 3 (87 : 13 *v*/*v*)	1	270	Plasma and vitreous fluid	[32]
RP-C18	Acetate buffer pH 3.5 : MeOH/triethylamine (82 : 18 v/v)	1	263	Goat plasma and milk	[33]
RP Ultrasphere XL-ODS C (75 × 4.6 mm I.D.)	20 mM AA pH 4 : 7% ACN	1	254	Human serum	[34]
Onyx Monolithic C18 (20 cm– 4.6 mm) coupled to Phenomenex C18 GC (5 cm 4.6 mm)	MeOH: 10 mM DPHP pH 7 (gradient)	1	254	Human plasma and dialysate	[35]
C18 with pre-C	NaOH buffer pH 3 : 1 M phosphoric acid: 0.01 Mn-octylamine pH 3.0 : ACN	1.3	259	Human urine	[36]
*μ*Bondapak C18 (30 cm × 3.9 mm × 10 *μ*m)	ACN: acetate buffer (5 : 95 *v*/*v*)	2	280	Plasma and dialysate-ultrafiltrate from patients	[37]
Supelcosil^TM^LC-18 (25 cm × 4.6 mm × 5 *μ*m), with a C18 GC	ACN: 0.075 M acetate buffer pH 5 (8 : 92, *v*/*v*)	0.8	230	Human plasma of burn patients	[38]
100 × 4.6 mm i.d. Perkin Elmer phenyl C (5 *µ*m)	ACN (including 0.015 M pentane sulfonic acid sodium pH 3.4 + glacial acetic acid and 4 with 45% KOH):water (5.5 : 94 *v*/*v*)	1.5	280	Aqueous solution	[39]
XTerra C18 (250 × 4.6 mm, 5 *μ*m) supported by Phenomenex C18 GC (4 × 3.0 mm)	MeOH : 40 mM phosphate buffer pH 3.2	1	260	Plasma and amniotic fluid	[40]
LiChrospher 100 RP C18 (250 mm × 4 mm, 5 lm particles)	MeOH: 10 mM phosphate buffer pH 7 (25 : 75 *v*/*v*)	1	256	Human serum, cerebrospinal fluid, and urine	[41]
C18	Acetate buffer pH 5.1: ACN: MeOH (5 : 20 : 75 v/v)	1	212	Pure and pharmaceutical dosage forms	[42]
Phenomenex ODS (4.6 × 250 mm, 5*µ*)	ACN : AA pH 4.9 : (8 : 92)	1.5	256	Pharmaceutical formulations	[43]
Acclaim 120 C18 (250 × 4.6 mm, 5 *μ*m particle size)	MeOH: sodium acetate buffer pH 6 (11 : 89 *v*/*v*)	1.8	220	Injections	[44]
Luna C18 (250 × 4.6 mm; 5 *μ*m)	Ethanol : water (45 : 55 *v*/*v*v)	0.5	258	Pharmaceutical dosage Form	[45]
C18 (250 × 25 mm) 25 *μ*m	Water: ACN (90 : 10 v/v)	1	212	CP in injections	[46]
Princeton-100 C18 (4.6 mm i.*d* × 250 mm., 5 *µ*n)	ACN: 25 mM PDPB pH 6.2 (6 : 9 4 *v*/*v*)	1	210	Bulk and pharmaceuticals	[47]
Hypersil Gold pentafluorophenyl (PFP) 6 (2.1 by 100 mm, 1.9 m)	(a) 10 mM phosphoric acid (b) ACN	0.5	260	Human plasma	[48]
C18	(ACN/0.1 M phosphoric acid/NaOH buffer pH 3): 0.01 M n-octylamine pH 3 (gradient)	1	256	Human urine	[49]

**Table 2:** Micellar electrokinetic chromatographic methods for determination of CP.

Technique	Column (C)	Mobile phase or eluent	Conditions	Matrices	Reference
MEKC	Uncoated FSC of 50 *μ*m	6 mM Na_2_B_4_O_7_, 10 mM Na_2_HPO_4_, 75 mM SDS pH 9.1	257^*∗∗*^, V of 15 kV	Human serum and plasma	[50]
MEKC	Uncoated FSC of 40.2 cm × 50 *μ*m id	Tris with SDS : MeOH	214^*∗∗*^, V of 15 kV	Plasma and cerebrospinal fluid	[51]
MEKC	Uncoated FSC of 31.2 cm (21 cm × 675 mm ID)	10 mM tris buffer pH 8.0 + 150 mM SDS and 20 mM tris buffer pH 9.0 + 200 mM SDS	254^*∗∗*^, V was 8 kV	Plasma and cerebrospinal fluid	[52]
MEKC	Bare FSC of 50 *µ*m, 5 mmol with length 56 cm	Imidazole buffer pH 5.1	240^*∗∗*^, V of 25 kV	NMP in CP for injection	[53]
MEKC	Uncoated FSC length 31.2 cm	Tris buffer + SDS as an electrolyte solution	214^*∗∗*^, V of 15 kV	Commercial injections	[54]
MEKC + indirect UV	MEKC [A 50 lm i.d 64.5 cm (56 cm detection length) bare FSC] IC [Gel IC-Cation-SW C (4.6 50 mm, 5 lm) supported by a water's cation GC (4.6·50 mm, 10 lm)]	MEKC (10 mM creatinine pH 3.8) IC (ACN: 0.01 mM nitric acid) (1 : 100)	225^*∗∗*^ MEKC (V of 30 kV) IC (1^*∗*^)	NMP in CP for injection	[55]
CZE	FSC (48.6 cm × 50 *µ*m i.d.) with 40.2 cm as a detection length 40.2 cm)	15 mm sodium borate buffer pH 9.3	215^*∗∗*^, V was 20 kV	Pharmaceutical formulations and human plasma	[56]

^*∗*^ (ml/min); ^*∗∗*^ (nm).

**Table 3:** Potentiometric and electrochemical methods for assay of CP.

Technique's name	Solvents/Conditions	Matrices	Reference
PH potentiometry	264 ^*∗∗*^ and 230^*∗∗*^ Dilution with UB (0.1 M CH_3_COOH + 0.1 MH_3_PO_4_ + 0.1 MH_3_BO_3_)	Pharmaceutical preparation	[57]
Electrochemical reduction and oxidation	WE (glassy carbon electrode), RE (AgCl), AE (platinum wire) The solutions were prepared in water and diluted with electrolytes	Pharmaceutical preparation	[58]
Electrochemical Reduction	A saturated AgCl (RE), WE (dropping mercury electrode), AE (glassy carbon) PB pH 2.7 (adjusted by 1 MH_3_PO_4_ + 1 M NaOH)	Pharmaceutical formulations and human urine samples	[59]
ASV + DPP	RE (Ag/AgCl/saturated KC), WE (dropping-mercury electrode), AE (platinum wire) For urine or plasma (PB pH 5.8), for serum (1 MH_3_PO_4_ and 1 M KOH pH 2.7) 0.1 M KCl used as ionic strength	Human urine, cerebrospinal fluid, and Serum	[60]

**Table 4:** Chromatographic technique with other techniques for determination of CP.

Technique	Column (C)	Mobile phase or eluent	Conditions	Matrices	Reference
R-HPLC-UV + (SPE)	C18	MeOH : ACN : AA	257^*∗∗*^ 0.9^*∗*^	Nutrient admixtures	[61]
LC	LiChrosorb RP-C18 (250 × 4.6 mm I.D., 5 *μ*m particle size)	MeOH : mM monosodium phosphoric acid pH 3 (13 : 87 v/v)	270^*∗∗*^ 1^*∗*^	The bile duct microdialysis probes	[62]
HILIC LC-MS/MS	HPLC Hypersil GOLD C (150 × 4.6 mm, 5 *μ*m) MS (spray voltage 3500 V, temperature 300°C, vaporizer temperature 400°C)	(a) 0.1% Formic acid:10 mM AA (b) 0.1% Formic acid:10 mM AA : MeOH (1 : 1 v/v) (c) 2-Propanol:acetone :ACN (1 : 1: 1 v/v/v)	Gas flow 6.5^*∗*^ Auxiliary gas flow 0.8^*∗*^	Plasma and cerebrospinal fluid	[63]
UPLC-MS/MS	RP Acquity BEH HILIC column (50 mm × 2.1 mm, 1.7 *μ*m, Waters)	(a) (ACN) (b) 20 mM AFB (Gradient)	0.5^*∗*^	Human plasma	[64]
(LC-GC-FID)	Extraction solvent (chloroform), SGE capillary C (30m × 0.25 mm)	Water : MeOH (12 : 88 v/v) : NaCl : carbonate/bicarbonate buffer pH 512	Flow rate 30^*∗*^ Hydrogen gas was used for the FID rate of air which was 300^*∗*^	NMP in CP (pharmaceutical preparation)	[65]
IC-SPE	Metrosep C4 4 mm × 250 mm cation exchange at 30°C	5% ACN:0.01 mlL^−1^ nitric acid	265^*∗∗*^	NMP in CP. HCl	[66]
SCX-LC/MS/MS	Zorbax300-SCX (2.1 mm × 50 mm, 5 *μ*m)	(a) ACN : 25 mM AFB pH 2.79 (5 : 95 v/v) (b) ACN : 500 mM AFB pH 2.79 + 25 mM AFB (30 : 70 v/v)	0.5^*∗*^ Curtain gas flow: 20psi; ion spray voltage: 5500 V; ion gas 1 and 2:	Mouse plasma	[67]
LC-MS/MS	Luna HILIC 200A, 100 × 2.0 mm, 3 *μ*m (Phenomenex) with a GC	ACN : 10 mM AFB pH 3.5 (72 : 28 v/v)	0.3^*∗*^	Plasma	[68]
HPLC-MS/MS	HPLC (Fortis reverse phase C8 (100 mm × 2.1 mm, 3 *μ*m)) MS (voltage 1.5 kV)	(a) Water-formic acid:10 mM AFB (0.1 : 99.9 v/v), B. MeOH	Gas flow rate, 600 l/h	Human serum	[69]
VAMS-LC/MS	Phenomenex (2.6 *μ*m, 100 Å, 50 × 4.6 mm)	(a) Water : 5 mM AA pH 5 (b) 5 mM AA in water : ACN (10 : 90 v/v)	0.5^*∗*^	Human whole blood	[70]
MEKC + UV + LC/MS	PFP Nucleodur HPLC column	MEKC (mM Na_2_B_4_O_7_ + 10 mM Na_2_HPO_4_ + 75 mM pH 9.1) HPLC ((a) 5 mM AFB pH 3, (b) 100% CAN)	254^*∗∗*^ 0.5^*∗*^	Urine	[71]
HPLC + MS	RP-C18	ACN : 10 mmolL^−1^ ammonium acetate (5 : 95)	0.8^*∗*^	Raw drug	[72]

**Table 5:** Spectrophotometric methods for the analysis of CP.

Technique's name	Solvent for dissolving and dilution	Conditions	Matrices	Reference
DRIR + XRD	8 ml of acetone was added as an eluent	Spectral limits 3587,3557 cm^−1^	Different hydrated forms of CP.2HCl	[73]
FTIR	The samples were diluted to 1000 mg with KBr Potassium bromide was used as a diluent	4000–400 cm^−1^	Pharmaceutical formulations	[74]
Savitzky–Golay differentiation filters and Fourier functions	Solutions prepared in concentration 100 *μ*g ml^−1^ in water	266^*∗∗*^	Human plasma	[75]
Complexation with Hg	Solutions were prepared in concentration 20–400 *μ*g ml^−1^ in water	257^*∗∗*^	Pharmaceutical dosage forms	[76]
Spectrophotometry with ammonium molybdate	Solutions were prepared in concentration 1000 *μ*g ml^−1^ in water	695^*∗∗*^	Pharmaceutical dosage forms	[77]
Spectrofluorometry		EXW (307), EMW (297), 435^*∗∗*^	Dosage forms	[78]
Spectrophotometry using a tetrazolium Salt	Solutions were prepared in concentration 20 *μ*g ml^−1^ with MeOH	483^*∗∗*^	Pharmaceutical dosage forms	[79]
UV spectrometry	Diluted with UB (0.1 M CH_3_COOH + 0.1 M H_3_PO_4_ + 0.1 M H_3_BO_3_)	264^*∗∗*^, 230^*∗∗*^	Pharmaceutical preparation	[57]
Fluorescence spectroscopy	Solutions were prepared with doubly distilled water	The EW was 280^*∗∗*^, 295^*∗∗*^The fluorescent intensity set at 341^*∗∗*^	Lysosome	[80]
UV + FTIR	Solutions were prepared in water; fluorescence intensity was measured in Tris/HCl solution pH 7.4	EW was 310^*∗∗*^ and EW set at 435^*∗∗*^	Pharmaceutical ingredient	[81]
Spectrophotometry	Solutions were prepared and diluted with 0.1 N NaOH	232^*∗∗*^	Pharmaceutical dosage forms	[82]
Spectrophotometry	Solutions were prepared and diluted with water	570^*∗∗*^	Pure and pharmaceutical dosage forms	[83]
Derivative spectrophotometry	Solutions were prepared and diluted with water	239, 254	Injections	[84]
Direct-infusion electrospray ionization	The solutions of NMP (N-methyl pyrrolidine) were prepared and diluted with water-MeOH (50 : 50)	ESI (V of 2000 V) flow of 7 l min^−1^, GOT of 250°C	NMP in CP	[85]
		FAIMS (V 75 and 375 V), electrode gaps (100 mm) with (700 mm) as a path length		
Microbiological assay	Powders were dissolved and diluted in water to give concentrations of 8.0, 16.0, and 32.0 *μ*g m^−1^	580^*∗∗*^	Injectable preparations	[86]

**Table 6:** Gas chromatographic methods for detection of CP.

Technique	Column (C)	Conditions	Matrices	Reference
GC	Wide-bore C (60m × 0.53 mm) coated with 100% polydimethylsiloxane (5 mm film)	Flow rate for CG 40, hydrogen 4 and air 100 ml/min	NMP in CP	[86]
		The sample was dissolved and diluted with chloroform		
		COT was 100°C, and the detector and the injector were 250°C		

## Abbreviations

CP: Cefepime
ACN: Acetonitrile
NaOH: Sodium hydroxide
KOH: Potassium hydroxide
MeOH: Methanol
PB: Phosphate buffer
PDPB: Potassium dihydrogen phosphate buffer
SDPM: Sodium dihydrogen phosphate monohydrate
C_40_H_84_BrN: Tetradecyl ammonium bromide
GC: Guard column
DPHP: Dibasic potassium hydrogen phosphate
AA: Ammonium acetate
SDS: Sodium dodecyl sulfate
MEKC: Micellar electrokinetic chromatography
CZE: Capillary zone electrophoresis
Na_2_HPO_4_: Disodium hydrogen phosphate
FSC: Fused-silica capillary
V: Voltage
ASV: Adsorptive stripping voltammetry
VAMS: Volumetric absorptive microsampling
DPP: Differential pulse polarography
AE: Auxiliary electrode
WE: Working electrode
RE: Reference electrode
SPE: Solid-phase extraction
LC/MS/MS: Liquid chromatography-tandem mass spectrometry
GC FID: Gas chromatography-flame ionization detection
UHPLC: Ultra-high-performance liquid chromatography
UPLC–MS/MS: Ultraperformance liquid chromatography-tandem mass spectrometry
SCX: High-performance hydrophilic strong cation exchange
HILIC LC-MS/MS: Interaction chromatography
IC-CD: Ion chromatography-conductivity detection
AFB: Ammonium formate buffer
AA: Ammonium acetate
GC: Gas Chromatography
CG: Carrier gas
COT: Column oven temperature
NMP: N-methylpyrrolidine
FTIR: Fourier transform infrared spectroscopy
EXW: Excitation wavelength
EMW: Emission wavelength.
